# Zhuye Shigao Decoction Combined with Qingqi Huatan Pills in Alleviating the Acute Exacerbation of Chronic Obstructive Pulmonary Disease (Phlegm-Heat Stagnating in the Lungs) via the IL-6-Mediated JAK1/STAT3 Signaling Pathway

**DOI:** 10.1155/2022/7942623

**Published:** 2022-05-06

**Authors:** Yunkun Chen, Wenbin Zhang

**Affiliations:** Department of Respiratory and Critical Care Medicine, Chongqing Traditional Chinese Medicine Hospital, No. 40, Daomenkou, Yuzhong District, Chongqing 400011, China

## Abstract

Chronic obstructive pulmonary disease (COPD) is a chronic disease with a long course which is often induced by an acute exacerbation of the disease by a respiratory tract infection. We aimed to explore the effect of Zhuye Shigao Decoction combined with Qingqi Huatan Pills on the regulation of the interleukin (IL)-6-mediated JAK1/STAT3 signaling pathway in rats with an acute exacerbation of COPD (phlegm-heat stagnating in the lungs). A model of COPD rats with lung phlegm-heat stagnation was established by smoking and intratracheal injection of lipopolysaccharide (LPS). The rats were randomly divided into eight groups: normal control, model control, three doses of herbs group, and three doses of herbs + itacitinib groups. The lung function indexes were measured by using a lung function tester, and changes in pathological features of all groups were observed by hematoxylin-eosin (HE) staining. The mRNA expression and protein expression levels in lung tissues were determined by real-time quantitative polymerase chain reaction (RT-qPCR), western blot, and immunohistochemical assay, respectively. Following treatment, IL-6 expression in lung tissues was significantly reduced compared with the model group. The results demonstrated that the medication was effective in alleviating the persistent airflow limitation and pathological features in COPD rats. Expression of JAK1/STAT3 in lung tissues was remarkably decreased. The JAK1/STAT3 pathway was inhibited, while SOCS3 expression was upregulated in the drug-treated groups compared with model control. However, after the addition of itacitinib (JAK1 inhibitor), the efficacy in each group was evidently impaired compared with herbs alone. Taken together, Zhuye Shigao Decoction combined with Qingqi Huatan Pills could improve the persistent airflow limitation and reduce lung inflammation and pathological changes of COPD possibly by regulating the expression of the IL-6-mediated JAK1/STAT3 pathway.

## 1. Introduction

Respiratory diseases cause a huge health burden worldwide. November 17, 2021, is World COPD Day. The Global Initiative for Chronic Obstructive Lung Disease (GOLD) has announced that COPD has affected 300 million people around the globe and has ended the lives of over 3 million people each year, making it the third leading cause of death worldwide [1].

COPD is a chronic inflammatory disease that progressively affects obstructive airflow limitation in the lungs. The manifestations include dyspnoea, coughing, coughing up mucus (sputum), and wheezing [2, 3]. This progressive airflow limitation eventually leads to airway remodeling and lung parenchymal destruction, and the progression of the disease is irreversible. In addition, the lung functions of COPD patients undergo a progressively abnormal decline and then chronic respiratory failure [4]. As one of the top three leading causes of death in China, the diagnostic rate varied from 23.61% to 30.00%. The medical cost ranged from 72 to 3,565 USD per year, accounting for 33.33% to 118.09% of the local average annual income [5]. Patients with COPD have been significantly impacted by health problems with poor quality of life (QOL).

Nevertheless, the pathogenesis of COPD has not yet been fully clarified. It is speculated that this disease is related to smoking, occupational dust, chemicals, air pollution, chronic inflammation of airway epithelial cells, enhanced oxidative stress response, imbalance of protease and antiprotease systems, and that the whole process is related to a multitude of cytokines and signal channels [6–8].

In temporary, the chronic inflammation mechanism of airway epithelial cells is universally accepted, involving a variety of inflammatory cells, cytokines, and inflammatory mediators. The Janus tyrosine kinase/signal transducer and activator of transcription (JAK1/STAT3) pathway plays an important role in the process of acute exacerbation of chronic obstructive pulmonary disease (AECOPD). It can mediate cell proliferation, differentiation, migration, apoptosis, and other biological reactions [9–11]. External stimuli either smoking or infection first activate airway epithelial cells to release massive inflammatory mediators, neutrophils, and macrophages. Meanwhile, additional inflammation-related cells in the body are accumulated in the airway in an active state allowing to accelerate the production of inflammatory mediators. Subsequently, more inflammatory cells are generated, recruited, and then combined with JAK receptors to activate the JAK1/STAT3 signaling pathway, triggering the acute COPD attack. In epithelial and immune cells, STAT3 serves as a key component of the JAK/STAT pathway. It can be activated by IL-6 intracellular, and then the expression of numerous proinflammatory genes in the lung is induced [12, 13]. The suppressors of cytokine signaling (SOCS3) can counteract interferon (IFN)-*γ*/STAT1 and IL-12/STAT4, IL-4/STAT6, growth hormone (GH)/STAT5, and IL-6/STAT3 [14]. In addition, SOCS3 has been identified as a negative feedback regulator of the JAK/STAT pathway [15] and has been demonstrated to be a target for inhibiting the activation of the JAK/STAT pathway in various inflammatory diseases [16].

Massive experimental studies have been conducted on the efficacy of traditional Chinese medicine (TCM) in the treatment of COPD-related signal transduction pathways, and findings have revealed that TCM treatment produces satisfactory effects on alleviating clinical symptoms and enhancing patients' physical fitness. It can also benefit patients with less number of attacks and a better quality of life, which is of important significance to the clinical study [4].

Some scholars have established a rat model of COPD and found that the percentage of pulmonary artery fiber, serum IL-6 content, and the expression of p-JAK2 and p-STAT3 are decreased after the intervention of Baofei Dingchuan Decoction, indicating that it can significantly reduce the weight of pulmonary blood vessels and improve lung functions of COPD rats [17].

Zhao Mei et al. have demonstrated the outstanding efficacy of Qingjin Huatan granules in the treatment of AECOPD with phlegm-heat stagnation. They have reported that AECOPD inflammation can be inhibited by downregulating p-STAT1, p-STAT3, p-JAK2, and JAK2 proteins and gene expression, and upregulating SOCS3 protein and gene expression [18]. Although there are various studies on JAK/STAT in TCM, there has been no research on the inflammatory response caused by the JAK1/STAT3 pathway mediated by IL-6.

This study intended to administer several doses of Zhuye Shigao Decoction combined with Qingqi Huatan Pills and different doses of herbs + itacitinib to intervene in the COPD rat model. The changes in lung function and lung tissue pathology were observed, and the expression of IL-6, JAK1, STAT3, and SOCS3 mRNA and proteins related to the JAK1/STAT3 pathway involved in chronic airway inflammation were determined. It is hypothesized that IL-6 initiated the expression of the STAT3 gene to mediate the inflammatory response caused by the JAK1/STAT3 pathway and promote the occurrence of AECOPD.

## 2. Materials and Methods

### 2.1. Animals

A total of 48 male specific-pathogen-free grade SD rats (6 for each group) weighing 200 ± 50 g and aged 10 to 12 weeks were purchased. All animals had adaptive feeding for 7 days in a clean and ventilated environment. The room temperature was set at 23 ± 2°C and atmosphere humidity at 60 ± 5%. Food and water were supplied ad libitum. The color of the fur, food intake, and behaviors were recorded.

### 2.2. Model Establishment and Grouping

The composition of Zhuye Shigao Decoction combined with Qingqi Huatan Pills included 15 g of light bamboo leaves, 30 g of raw gypsum, 15 g of French *Pinellia*, 20 g of *Ophiopogon japonicus*, 10 g of ginseng, 6 g of licorice, 10 g of scutellaria, 30 g of melon seeds, 12 g of dannan star, 15 g of tangerine peel, 10 g of bitter almonds, 15 g of *Citrus aurantium*, 30 g of *Houttuynia cordata*, 10 g of Bulbus Fritillariae Thunbergii, and 15 g of Zhuru. All of the herbs were purchased from the Department of Pharmacy at the Chongqing Hospital of Traditional Chinese Medicine and produced by Sichuan Kangmei Pharmaceutical to ensure experimental results were reliable. According to the dosage of medication, the animals were divided into low (5 g·kg^−1^/d), medium (10 g·kg^−1^/d), and high-dose (15 g·kg^−1^/d) intervention groups. The dosage was determined based on our previous study and the published literature of modern medical laboratory zoology [19, 20]. Each drug was prepared according to the specific dosage, dissolved in distilled water, and finally adjusted to a crude drug amount of 2 g/mL.

The COPD model of rats was induced by cigarette smoke combined with lipopolysaccharide after 1 week of adaptive feeding [21]. There were eight groups with six rats in each one: normal control, model control, three doses of herbs group, and three doses of herbs + itacitinib group according to the weight based on the random number table method. The different doses of herbs with or without itacitinib (30 mg/kg) were administered by gavage and subcutaneous injection, respectively. Apart from the normal control group (NC), on the 1^st^ and 14^th^ days, all rats were anesthetized with 4% pentobarbital sodium and the tracheas were exposed to 200 *μ*L of lipopolysaccharide (LPS, 1 g/mL). Rats were placed into a 50 cm × 40 cm × 40 cm glass smoked poisoning box and exposed to the smoke from the ignition of an appropriate amount of sawdust and 20 cigarettes mixture from day 2 to 30. The rats were exposed to smoke twice per day (30 min each time) and rested two days a week to establish the experimental model. After the COPD model was successfully established, the herbal treatment with or without itacitinib was given to the rats for 14 consecutive days, while the NC and model control were given equal saline.

### 2.3. Histopathology

The right lung tissue of rats was fixed with 4% formaldehyde, routinely embedded in paraffin and cut into 5 *μ*m serial sections. The sections were then progressively dewaxed with xylene, dehydrated with ethanol, stained with eosin and hematoxylin, and sealed with neutral gum. The morphological changes of the bronchus and lung tissues were observed under a light microscope and analyzed (Jetta Company, Shanghai, China).

### 2.4. Immunohistochemistry

Immunohistochemistry (IHC) analysis was carried out by using MaxVisionTM techniques (Maixin Bio, China) based on the manufacturer's instructions. Firstly, the lung tissue was fixed by 4% paraformaldehyde (Solarbio, Shanghai, China), dehydrated, and paraffin embedded. The 5 *μ*m thick slides were obtained. The deparaffinization and hydration were performed, the slides were then incubated with 3% H_2_O_2_ (Sinopharm, China) for 10 min and 0.1% trypsin (Beyotime, China) for 20 min. The primary antibodies were incubated at 4°C overnight and then incubated with HRP-polymer-conjugated secondary antibodies at 37°C for 1 h. The slides were then stained by using the chromogenic reagent diaminobenzidine (DAB, Zhongshan, Beijing, China) for 3 min and counterstained with hematoxylin (Jiancheng, Nanjing, China). An inverted microscope (Olympus, Japan) was employed for image acquisition. The primary antibodies anti-IL-6, anti-JAK1, anti-STAT3, and anti-SOCS3 were purchased from Cell Signaling Technology (CST).

### 2.5. ELISA Assay

The rats were anesthetized by intraperitoneal injection of 4% sodium pentobarbital. The serum of each group was collected. The sample was taken at −80°C and prepared in advance. The detection was performed strictly according to the instructions of the ELISA kit manufacturer (R&D Systems, Emeryville, CA, USA). Firstly, the diluted primary antibody was added to the appropriate wells and incubated for 2 h at room temperature. A blocking solution of 300 *µ*L was added to each well and incubated for 1 h at room temperature after three cycles of washing with 0.05% Tween-20. Then, the plate was washed twice with a wash solution. The diluted biotinylated detection antibody was added and incubated for 1 h at 37°C, and the plate was washed three times. Subsequently, 100 *µ*L of diluted AKP conjugated streptavidin was added and incubated for 1 h at room temperature. The plate was emptied and washed three times for a total of 15 min and washed five more times. The substrate was collected for color development for 30 min at room temperature. Finally, 0.05 mL of 2 M of H_2_SO_4_ was added to each well and immediately read with a plate reader at 405–410 nm.

### 2.6. Quantification of mRNA

The expression quantification of IL-6, JAK1, STAT3, and SOCS3 mRNA in rat lung tissue was detected by reverse transcription quantitative real-time polymerase chain reaction (RT-PCR) technology. The lung tissue was collected, and total RNA was extracted from the tissue by the TRIzol method. The subsequent reverse transcription into cDNA was performed using Superscript II RT (Invitrogen, China). cDNA was amplified by adding equivalent amounts of initial RNA quantity to the reaction mix including 12.5 *μ*L of SYBR Green (Invitrogen), forward and reverse primers (10 pmol/ml), with 0.5 *μ*L for each primer, and nuclease-free water to final volumes of 25 *μ*L per well. Relative fold changes were quantified using the 2^−△△^Ct formula. Primers used were as follows: IL-6-F, 5′- CTCCCAACAGACCTGTCTATAC-3′; IL-6-R, 5′- CCATTGCACAACTCTTTTCTCA-3′; JAK1-F, 5′-TCTGTTTGCTCAGGGACAGT-3′; JAK1-R, 5′- AGCCATCCCTAGACACTCGT-5′; STAT3-F, 5′- ATCACGCCTTCTACAGACTGC-3′; STAT3-R, 5′- CATCCTGGAGATTCTCTACCACT-3′; SOCS3-F, 5′- CCTGCGCCTCAAGACCTTC-3′; SOCS3-R, 5′- GTCACTGCGCTCCAGTAGAA-3′; GAPDH-F, 5′-AGGTCGGTGTGAACGGATTTG-3′; and GAPDH-R, 5′-TGTAGACCATGTAGTTGAGGTCA-3′.

### 2.7. Western Blot

The western blot (WB) assay was used to detect the expression changes of STAT1 and STAT3 in rat lung tissues. Stored rat lung tissues were lysed using RIPA reagent (Beyotime, China), prepared and detected using protein gel electrophoresis. Proteins were transferred to a PVDF membrane, blocked, and incubated with diluted primary antibody, and then secondary antibody. The primary and secondary antibodies were incubated for 1 h and 1–2 h, respectively. Protein visualization was conducted using an enhanced chemiluminescence detection kit (Solarbio, China). The Image J 1.8.0 software was used to determine the optical density values of protein bands and the internal control *β*-actin, and the relative density of the protein in each group was calculated from the ratio of the two. Immunoblotting was performed and blots were probed with antibodies against IL-6, JAK1, STAT3, SOCS3, and *β*-actin (CST, USA).

### 2.8. Statistical Analysis

Statistical analysis was performed using GraphPad Prism software, version 8.0.1. The data were reported as the mean ± standard error (SD). Differences between groups were analyzed using one-way ANOVA with Tukey analysis of variance for comparison of more than two groups. *P* values of <0.05 were considered statistically significant.

## 3. Results

### 3.1. The IL-6 Expression in Lung Tissue Is Inhibited

Various methodologies were used to detect the expression of IL-6 in lung tissues. The results of immunohistochemical experiments are shown in Figure 1(a). Compared with NC, the number of brown-positive cells in MC was significantly increased. Compared with MC, the positive cells in the herbs intervene group were significantly reduced, and the decline was most significant in the high-dose herbs group. Itacitinib was utilized to block the JAK-STAT3 pathway transduction. In medium- and high-dose herbs + itacitinib groups, the positive cells were decreased compared with the MC but increased evidently compared with the corresponding herbs treated group. However, no apparent decrease in the number of positive cells was observed in the low-dose herbs + itacitinib group. In addition, WB was used to detect the expression of IL-6 protein, and semiquantitative analysis was performed based on the gray value, as shown in Figure 1(c). It is revealed that the expression of IL-6 was upregulated in the model group, and the expression of IL-6 could be significantly downregulated in the herbs intervention group. While IL-6 expression was increased in herbs + itacitinib groups compared with herb groups; however, it was still lower than the model control. Moreover, the gene expression was detected using RT-qPCR, and the expression trend was consistent with immunohistochemistry and WB results (Figure 1(b)).

### 3.2. The Lung Function Is Improved and Pathological Changes in Lung Tissues Are Reduced

The peak inspiratory flow (PIF), peak expiratory flow (PEF), and minute ventilation volume (MV) were measured for detecting lung functions of rats, as shown in Figure 2, compared with NC, PIF, PEF, and MV were decreased significantly in MC, indicating airflow limitation, pulmonary ventilation dysfunction, and successful COPD modeling. The values of PIF, PEF, and MV in the herbs treated group were increased remarkably in contrast to MC. The value of PIF in the herbs + itacitinib groups was also increased markedly (Figure 2(a)), whereas those of PEF and MV were increased only in the medium- and high-dose herbs + itacitinib groups (Figures 2(b) and 2(c)). Compared with the herbs + itacitinib groups, the PIF and MV values of the herbs group were significantly higher than the corresponding dose intervention groups (*P* < 0.05), and the PEF value was also increased, but there were no statistics in the low-dose herbs group. These findings demonstrated that all doses of herbs could improve lung airflow limitation and ventilatory dysfunction, and the improvement effect on lung function was significantly reduced after inhibiting JAK-STAT3 signal transduction.

The changes in lung tissue histopathology were observed using HE staining. The lung tissue of the rats in NC was clearly visible, and the bronchial wall structure was relatively regular, without obvious damage. Only a small infiltration of inflammatory cells was seen, mucus plugs and mucus were not observed, and the congestion and edema of the mucous membrane were not observed (Figure 2(d)). The lung tissue of MC showed glandular hyperplasia in multiple locations, a large number of inflammatory cells were infiltrated, and the tube wall thickened. The structure of the alveolar wall was severely damaged, thinned, and broken, allowing the formation of pulmonary bullae, and the number of alveoli was reduced. Compared with MC, the lung tissue pathology in the herbs mid and high groups was significantly attenuated. The bronchial wall thinning, partial shedding, inflammatory cell infiltration, congestion, and edema were alleviated, and pulmonary bullae were reduced. And the destruction of the alveolar cavity, expansion, and fusion were eased. In the herbs low + itacitinib group, the lung tissue pathology was not significantly improved compared with the herbs intervention groups. While the alveolar expansion and fusion, inflammatory cell infiltration, and mucosal congestion were improved in the herbs mid + itacitinib group. Moreover, the pathological improvement of the herbs high + itacitinib group was better than that of the herbs mid + itacitinib group.

### 3.3. Changes in Serum Cytokine Levels

The rat serum was collected for ELISA and the results are shown in Figure 3. The serum levels of IFN-*γ*, IL-4, IL-4R, IL-12, and IL-12R in MC were significantly increased compared with NC. Compared with the MC, the levels of IFN-*γ*, IL-4, IL-4R, IL-12, and IL-12R in the serum of rats in each dose group of herbs decreased remarkably, and the herbs high group had the strongest effect. The cytokine content in the herbs + itacitinib group increased compared with different doses of herbs groups. It was found that all dose groups of herbs were effective in reducing serum inflammatory factors in COPD model rats, and the high-dose group produced the best effect, while the ability of herbs to decrease serum inflammatory factors in the herbs + itacitinib group was reduced.

### 3.4. Expression of the JAK1/STAT3 Signaling Pathway in Lung Tissues

The results of the immunohistochemistry experiment are shown in Figure 4(a). The number of JAK1 brown-positive cells in the lung tissue sections of the MC was increased significantly compared with NC. Compared with MC, the number of positive cells in the herbs treatment was significantly reduced, most notably in the high-dose group. After the addition of itacitinib to inhibit the JAK-STAT3 pathway, positive cells in the herbs mid and high + itacitinib groups were lower than those in the MC, while in the herbs low + itacitinib group, no significant decline in the number of positive cells was observed. WB was subsequently employed to detect the expression of JAK1 and STAT3 proteins and semiquantitatively analyzed based on the gray value, as shown in Figures 4(b), 4(d), and 4(f), and the expression of JAK1 and STAT3 was increased in the MC, and the difference was significant. The herbs could significantly downregulate JAK1 and STAT3 expression. After the JAK-STAT3 was blocked by itacitinib, the expression of JAK1 and STAT3 was increased in each dose group of herbs compared with the corresponding herbs dose of the itacitinib-free group, and the difference was significant. In addition, the immunohistochemical staining results of STAT3 are shown in Figure 4(e). RT-qPCR showed that compared with the NC, the expression of JAK1 and STAT3 mRNA in the lung tissue of rats was significantly increased in the model control. Herbs treatment could significantly reduce the expression of JAK1 and STAT3 mRNA levels. After the interference of JAK1 inhibitor itacitinib, the JAK1 and STAT3 mRNA expression of the herbs treated group was increased remarkably (Figures 4(c) and 4(g)).

### 3.5. SOCS3 Expression Is Upregulated in Lung Tissue

SOCS3 protein expression in rat lung tissue was detected by WB and IHC (Figure 5(a)–5(c)). The SOCS3 brown positive cells in the lung tissue sections of the MC were significantly reduced (Figure 5(b)). Compared with the MC, the number of positive cells in the herb mid and high groups was significantly increased. In the herbs + itacitinib group, there was no significant change in the number of positive cells compared with the MC, except for the herbs high + itacitinib group. The expression of SOCS3 mRNA in lung tissue was detected by RT-qPCR which was significantly reduced in MC (Figure 5(d)). The herbs treatment could significantly increase the expression of SOCS3 mRNA. In the presence of itacitinib, SOCS3 mRNA in each herbs dose group decreased, and there was no significant difference in herbs low and mid group compared with MC (Figure 5(d)).

## 4. Discussion

COPD is one of the common respiratory diseases in the clinic which is mostly characterized by continuous airflow limitation, and seriously affects the quality of life and safety of patients [22]. The inducing factors are mainly related to the chronic inflammatory reaction of the airway and lung tissue caused by harmful gases or particles in the environment, and they are the continuous airway inflammatory reaction. COPD airway inflammation involves all airways and lung tissues, involving macrophages, neutrophils, IL-8, TNF-ɑ, cytokines, and inflammatory mediators [23, 24]. Inflammatory factors play a dominant role in the occurrence and development of COPD, and IL-6 is an important proinflammatory factor in the complex inflammatory cell-cytokine network in the airway inflammation of COPD. Studies have shown that IL-6 is elevated to various degrees in sputum, lung parenchyma, and blood in COPD patients [25, 26]. Continuous activation and overexpression of STAT1 and STAT3 in airway epithelial cells are closely related to airway inflammation [27], which is widely involved in mediating the expression and regulation of inflammatory cytokines. The study has reported that several inflammatory cells can release inflammatory factors and inflammatory chemokines under the COPD mechanism and participate in cell proliferation, differentiation, apoptosis, inflammatory response, and other pathophysiological mechanisms through the JAK/STAT signaling pathway [28].

In this experiment, the COPD model rats were prepared by combining smoking and LPS, using different doses of TCM Zhuye Shigao Decoction combined with Qingqi Huatan Pills to gavage rats. It was found that each dose group of herbs could improve the lung function of rats' PIF, PEF, and MV, and relieve lung airflow limitation and ventilatory dysfunction, thereby alleviating lung tissue disease and bronchial wall inflammation. It was also confirmed that IL-6, JAK1, and STAT3 mRNA and protein were significantly highly expressed in COPD rats, indicating that the occurrence and development of COPD were closely related to the continuous activation and overexpression of JAK1/STAT3 and abnormal signal transduction pathways in lung tissues, and the activation level of STAT3 was closely and positively correlated to IL-6. It is reported that cytokines play a role in regulating gene transcription by acting on cell surface receptors by activating signal transducers, that is, sending out a series of signal molecules and transmitting the stimulating signal to the target gene in the nucleus. The expression of the proinflammatory factor IL-6 was significantly increased under the combined induction of smoking and LPS. IL-6R on the cell surface was combined, further inducing phosphorylation of JAK1. JAK1 activation quickly combines with STAT3 to phosphorylate STAT3 and activate it. STAT3 could regulate the transcription and expression of related genes. The TCM Zhuye Shigao Decoction combined with Qingqi Huatan Pills could reduce the expression of IL-6, JAK1, and STAT3 mRNA and protein in lung tissues and inhibit the serum cytokines IFN-*γ*, IL-4, IL-4R, IL-12, and IL-12R. T cells secreting IFN-*γ* in the airways of COPD patients increase, and IFN-*γ* levels in patients with COPD were increased. IFN-*γ* coordinates the infiltration of T cells in COPD lungs by upregulating CXC-chemokine receptor (CXCR) 3 on these cells and the release of chemokines that activate CXCR3 [29]. Previous studies have found that IL-4 and IL-12 are significantly elevated in AECOPD patients [30]. By using itacitinib for JAK-STAT3 pathway intervention, compared with their corresponding doses of itacitinib free groups, the expressions of IL-6, JAK1, and STAT3 mRNA and protein in the lung tissue of each dose group of herbs were significantly increased, and serum IFN-*γ*, IL- 4, IL-4R, IL-12, and IL-12R also increased significantly.

Cytokines are important factors in the JAK/STAT signaling pathway, which are transmitted from the cell membrane to the nucleus, and the inhibitor of cytokine transduction (SOCS) is transduced by the JAK/STAT signal and has a negative regulatory effect by specifically negatively regulating the induction and activation of the JAK/STAT pathway [31]. SOCS3 is activated to negatively regulate the JAK/STAT pathway, and it is generally believed that SOCS3 is the target gene of STATs and can directly inhibit the activation of STATs at present [32]. WB, IHC, and RT-qPCR assays were used to detect the expression of SOCS3 in lung tissues. The results showed that Zhuye Shigao Decoction combined with Qingqi Huatan Pills could significantly increase the SOCS3 expression of mRNA and protein in lung tissues. In contrast to the corresponding itacitinib free Herbs intervention group, the expression of SOCS3 mRNA and protein in the lung tissue of the herbs group in the presence of itacitinib was significantly reduced.

## 5. Conclusions

The described results revealed that Zhuye Shigao Decoction combined with Qingqi Huatan Pills could alleviate the continuous airflow limitation of COPD and reduce lung inflammation and pathological changes. It has been demonstrated that the herbs can downregulate the overexpression and continuous activation of JAK1 and STAT3 in the JAK/STAT signaling pathway based on IL-6 and upregulate SOCS3 to negatively regulate JAK/STAT signals, thereby inhibiting the AECOPD attack. In addition, JAK/STAT3 can be used as the main target for the treatment of COPD patients that are overactivated by JAK/STAT3. Further research after the intervention of TCM will provide basic support for the treatment of AECOPD with TCM and prevent its occurrence and development. However, the study was short of methodology on molecular mechanism exploration and was limited to the COPD rat investigation. Moreover, the herbs' adverse effects were not investigated. Subsequent research is needed to mainly focus on the limitations mentioned above.

## Figures and Tables

**Figure 1:** IL-6 expression is inhibited in lung tissues. (a) The photomicrographs of immunohistochemical staining for IL-6 among lung tissue samples are displayed. The nucleus is colored in blue and the positive cells are colored in brown (scale bar is 50 *µ*m, ×400). (b) The relative IL-6 gene expression. (c) Western blot analysis of IL-6 in lung tissues. Each group in the strip chart is consistent with the below semiquantitative analysis on the basis of the intensity of the strip chart. Error bars represent SD, *n* = 3. ^*∗*^, ^#^, ^&^, and ^Δ^ represent *P* values <0.05 which are considered statistically significant. ^*∗*^ versus MC (model control), ^#^ versus herbs low, ^&^ versus herbs mid, and ^Δ^ versus herbs high.

**Figure 2:** Zhuye Shigao Decoction combined with Qingqi Huatan Pills is able to improve lung function and alleviate pathological changes in lung tissue. (a) PIF, (b) PEF, and (c) MV detection as shown in the diagram. (d) HE staining for the lung tissue of SD rats (scale bar is 50 *µ*m, ×400). Error bars represent SD, *n* = 3. ^*∗*^, ^#^, ^&^, and ^Δ^ represent *P* values <0.05 which are considered statistically significant. ^*∗*^ versus MC (model control), ^#^ versus herbs low, ^&^ versus herbs mid, and ^Δ^ versus herbs high.

**Figure 3:** Cytokines level in serum is detected by ELISA. (a) IFN-*γ* concentration in serum. (b) IL-4, IL-4R, IL-12, and IL-12R were measured by ELISA. Error bars represent SD, *n* = 3. ^*∗*^, ^#^, ^&^, and ^Δ^ represent *P* values <0.05 which are considered statistically significant. ^*∗*^ versus MC (model control), ^#^ versus herbs low, ^&^ versus herbs mid, and ^Δ^ versus herbs high.

**Figure 4:** Expression of the JAK1/STAT3 signaling pathway of lung tissue in each group. (a) JAK1 protein expression of lung tissue detected by immunohistochemistry is presented by photomicrographs. The nucleus is colored in blue and the positive cells are colored in brown (scale bar is 50 *µ*m, ×400). (b) The strip chart of JAK1 and STAT3, *β*-actin was used as the internal reference. (c) The relative JAK1 gene expression. (d) Semiquantitative analysis based on the intensity of strip chart for JAK1 in lung tissue. (e) STAT3 protein expression of lung tissue detected by immunohistochemistry was presented by photomicrographs. The nucleus is colored in blue and the positive cells are colored in brown (scale bar is 50 *µ*m, ×400). (f) Semiquantitative analysis of STAT3 expression. (g) Gene expression of STAT3. Error bars represent SD, *n* = 3. ^*∗*^, ^#^, ^&^, and ^Δ^ represent *P* values <0.05 which are considered statistically significant. ^*∗*^ versus MC (model control), ^#^ versus herbs low, ^&^ versus herbs mid, and ^Δ^ versus herbs high.

**Figure 5:** SOCS3 expression is upregulated in lung tissue. (a) Western blot analysis of SOCS3 in lung tissue, *β*-actin was used as the internal reference. (b) The photomicrographs of immunohistochemical staining for SOCS3 among lung tissue samples are displayed. The nucleus is colored in blue and the positive cells are colored in brown (scale bar is 50 *µ*m, ×400). (c) Semiquantitative analysis on the basis of the intensity of protein bands in eight groups. (d) The relative SOCS3 gene expression. Error bars represent SD, *n* = 3. ^*∗*^, ^#^, ^&^, ^Δ^ represent *P* values <0.05 which are considered statistically significant. ^*∗*^ versus MC (model control), ^#^ versus herbs low, ^&^ versus herbs mid, and ^Δ^ versus herbs high.

## Data Availability

The data used to support the findings of this study are included within the article.

## References

[1] Global Strategy for Prevention (2020). Diagnosis and management of COPD. https://goldcopd.org/gold-reports/.

[2] Kukrety S. P., Parekh J. D., Bailey K. L. (2018). Chronic obstructive pulmonary disease and the hallmarks of aging. *Lung India: Official Organ of Indian Chest Society*.

[3] Joshi M., Varkey B. (2019). Editorial. *Current Opinion in Pulmonary Medicine*.

[4] Lange P., Celli B., Agustí A. (2015). Lung-function trajectories leading to chronic obstructive pulmonary disease. *New England Journal of Medicine*.

[5] Zhu B., Wang Y., Ming J., Chen W., Zhang L. (2018). Disease burden of COPD in China: a systematic review. *International Journal of Chronic Obstructive Pulmonary Disease*.

[6] Lv X.-X., Liu S.-S., Li K., Cui B., Liu C., Hu Z.-W. (2017). Cigarette smoke promotes COPD by activating platelet-activating factor receptor and inducing neutrophil autophagic death in mice. *Oncotarget*.

[7] Chen J., Dai L., Wang T., He J., Wang Y., Wen F. (2019). The elevated CXCL5 levels in circulation are associated with lung function decline in COPD patients and cigarette smoking-induced mouse model of COPD. *Annals of Medicine*.

[8] Yang M., Kohler M., Heyder T. (2018). Proteomic profiling of lung immune cells reveals dysregulation of phagocytotic pathways in female-dominated molecular COPD phenotype. *Respiratory Research*.

[9] Yew-Booth L., Birrell M. A., Lau M. S. (2015). JAK-STAT pathway activation in COPD. *European Respiratory Journal*.

[10] Kuusanmäki H., Dufva O., Parri E. (2017). Drug sensitivity profiling identifies potential therapies for lymphoproliferative disorders with overactive JAK/STAT3 signaling. *Oncotarget*.

[11] Wang C., Li Z., Liu X. (2015). Effect of liuweibuqi capsule, a Chinese patent medicine, on the JAK1/STAT3 pathway and MMP9/TIMP1 in a chronic obstructive pulmonary disease rat model. *Journal of Traditional Chinese Medicine*.

[12] Huan W., Tianzhu Z., Yu L., Shumin W. (2017). Effects of ergosterol on COPD in mice via JAK3/STAT3/NF-*κ*B pathway. *Inflammation*.

[13] Naugler W. E., Karin M. (2008). The wolf in sheep’s clothing: the role of interleukin-6 in immunity, inflammation and cancer. *Trends in Molecular Medicine*.

[14] Dalpke A., Heeg K. (2003). Suppressors of cytokine signaling proteins in innate and adaptive immune responses. *Archivum Immunologiae et Therapiae Experimentalis*.

[15] Chaves de Souza J. A., Nogueira A. V., Chaves de Souza P. P. (2013). SOCS3 expression correlates with severity of inflammation, expression of proinflammatory cytokines, and activation of STAT3 and p38 MAPK in LPS-induced inflammation in vivo. *Mediators of Inflammation*.

[16] Suzuki A., Hanada T., Mitsuyama K. (2001). Cis3/Socs3/Ssi3 plays a negative regulatory role in Stat3 activation and intestinal inflammation. *Journal of Experimental Medicine*.

[17] He F., Shen Y., Xu J. (2017). Effect of Baofei dingchuan decoction on JAK/STAT signal transduction pathway of pulmonary artery in rats with chronic obstructive pulmonary disease. *Journal of Traditional Chinese Medicine*.

[18] Zhao M., Xu G., Li J. (2019). Effect of qingjin huatan granule on JAK/STAT signal pathway in lung tissue of rats with chronic obstructive pulmonary disease in acute exacerbation stage. *Journal of Traditional Chinese Medicine*.

[19] Wen-bin Z., Wen-hui L., Ying-kai F. (2017). Add and subtract therapy of Zhuye Shigao decoction combined with Qingqi huatan Pills on chronic obstructive pulmonary disease at acute and aggravating period. *Chinese Journal of Experimental Traditional Meddicine Formula*.

[20] Shi X. (2000). *Xiandai Yixue Shiyan Dongwuxue [M]*.

[21] Lin D., Li S., Hou C., Xu X., Guo S., Wang Q. (2021). Exploring the biological mechanism of qi deficiency syndrome with chronic obstructive pulmonary disease (COPD) based on integrated pharmacology. *Journal of Traditional Chinese Medical Sciences*.

[22] Tulic M. K., Piche T., Verhasselt V. (2016). Lung-gut cross-talk: evidence, mechanisms and implications for the mucosal inflammatory diseases. *Clinical and Experimental Allergy*.

[23] Victoni T., Barreto E., Lagente V., Carvalho V. F. (2021). Oxidative imbalance as a crucial factor in inflammatory lung diseases: could antioxidant treatment constitute a new therapeutic strategy?. *Oxidative Medicine and Cellular Longevity*.

[24] Beasley V., Joshi P. V., Singanayagam A., Molyneaux P. L., Johnston S. L., Mallia P. (2012). Lung microbiology and exacerbations in COPD. *International Journal of Chronic Obstructive Pulmonary Disease*.

[25] Xu H., Shi X., Li X. (2020). Neurotransmitter and neuropeptide regulation of mast cell function: a systematic review. *Journal of Neuroinflammation*.

[26] Caetano M. S., Zhang H., Cumpian A. M. (2016). IL6 blockade reprograms the lung tumor microenvironment to limit the development and progression of K-ras-mutant lung cancer. *Cancer Research*.

[27] Gong J. H., Shin D., Han S. Y. (2013). Blockade of airway inflammation by kaempferol via disturbing tyk-STAT signaling in airway epithelial cells and in asthmatic mice. *Evid Based Complement Alternat Med*.

[28] Jenkins B. J. (2014). Transcriptional regulation of pattern recognition receptors by JAK/STAT signaling, and the implications for disease pathogenesis. *Journal of Interferon and Cytokine Research*.

[29] Mitra A., Vishweswaraiah S., Thimraj T. A. (2018). Association of elevated serum GM-CSF, IFN-*γ*, IL-4, and TNF-*α* concentration with tobacco smoke induced chronic obstructive pulmonary disease in a south Indian population. *International Journal of Inflammation*.

[30] Wei B., Sheng Li C. (2018). Changes in Th1/Th2-producing cytokines during acute exacerbation chronic obstructive pulmonary disease. *Journal of International Medical Research*.

[31] Uren R. T., Turnley A. M. (2014). Regulation of neurotrophin receptor (Trk) signaling: suppressor of cytokine signaling 2 (SOCS2) is a new player. *Frontiers in Molecular Neuroscience*.

[32] Li X. D., Li X. M., Gu J. W., Sun X. C. (2020). MiR-155 regulates lymphoma cell proliferation and apoptosis through targeting SOCS3/JAK-STAT3 signaling pathway [J]. *European Review for Medical and Pharmacological Sciences*.

